# A novel gemycircularvirus in an unexplained case of child encephalitis

**DOI:** 10.1186/s12985-015-0431-0

**Published:** 2015-11-24

**Authors:** Chenglin Zhou, Shibing Zhang, Qin Gong, Aimin Hao

**Affiliations:** Department of Laboratory Medicine, Jiangsu Taizhou People’s Hospital, Taizhou, Jiangsu 225300 China; Department of Laboratory Medicine, the First People’s Hospital of Suqian, Suqian, Jiangsu 223800 China; Jiangsu Taizhou People’s Hospital, Taizhou, Jiangsu 225300 China; Department of Laboratory Medicine, the Second People’s Hospital of Wuxi, Wuxi, Jiangsu 214002 China

**Keywords:** Gemycircularvirus, Unexplainable encephalitis, Complete genome

## Abstract

**Background:**

Recently, a diverse group of viruses with circular, replication initiator protein(Rep) encoding, single stranded DNA (CRESS-DNA) genomes, were discovered from wide range of eukaryotic organisms ranging from mammals to fungi. Gemycircularvirus belongs to a distinct group of CRESS-DNA genomes and is classified under the genus name of Gemycircularvirus.

**Findings:**

Here, a novel gemycircularvirus named GeTz1 from cerebrospinal fluid sample of a child with unexplainable encephalitis was characterized. The novel gemycircularvirus encodes two major proteins, including a capsid protein (Cap) and a replication-associated protein (Rep). Phylogenetic analysis based on the amino acid sequence of Rep indicated that GeTz1 clusters with one gemycircularvirus discovered from bird (KF371633), sharing 46.6 % amino acid sequence identity with each other.

**Conclusion:**

A novel gemycircularvirus was discovered from cerebrospinal fluid sample of a child with unexplainable encephalitis. Further studies, such as testing human sera for specific antibodies, should be performed to investigate whether gemycircularvirus infects human and is associated with encephalitis.

## Findings

Viruses with small circular ssDNA genomes include a diverse group of viruses with circular, replication initiator protein(Rep) encoding, single stranded DNA (CRESS-DNA) genomes, and can infect a wide range of eukaryotic organisms ranging from mammals to fungi [1]. Recent reports discovering CRESS-DNA genomes including from cerebrospinal fluid (CSF) from patients with encephalitis suggested their potential associations with encephalitis [2–6]. Gemycircularvirus belongs to a distinct group of CRESS-DNA genomes which is classified under the proposed genus name of Gemycircularvirus [7, 8]. The members of this proposed genus are also called myco-like viruses because their overall genome shows similar to that of Sclerotinia sclerotiorum hypovirulence-associated DNA virus 1 (SsHADV-1), which is the first member of gemycircularvirus genus and found in fungi [9]. Then the gemycircularvirus genomes were subsequently identified in feces of different animals [8, 10], plant [11–13], the body of insects [7, 14], and sewage [8, 15]. Gemycircularviruses were also recently reported in blood from a patient with multiple sclerosis [16], and in the cerebrospinal fluid (CSF) of encephalitis patients [3]. Here, using sequence-independent PCR amplification and sequence similarity searches, we detected gemycircularvirus in the CSF of an encephalitic child, China.

Within 2014, 20 CSF samples were obtained from children (<6 years old) with encephalitis. All of these samples were tested negative for known pathogens (including virus, bacteria and parasite) at the Division of Clinical Microbiology of Taizhou People’s Hospital. Ethical Approval was given by Ethics Committee of Taizhou People’s Hospital and the reference number is No. TZYXLL2015033. In order to investigate whether these cases of encephalitis were caused by viruses, sequence-independent PCR amplification as previously described [17] was used. During the whole process of sequence-independent PCR amplification, 21 individual samples including 20 CSF samples and 200 microliters of phosphate-buffered saline (PBS) as a negative control were studied separately and parallel. Briefly, 200 microliters of each sample was collected after centrifugation (10 min, 15,000 × *g*) and filtered through a 0.45-μm filter (Millipore) to remove eukaryotic and bacterial cell-sized particles. The filtrates enriched in viral particles were treated with a mixture of DNases (Turbo DNase from Ambion, Baseline-ZERO from Epicentre, and benzonase from Novagen) and RNase (Fermentas) to digest unprotected nucleic acid at 37 °C for 60 min [18]. Viral nucleic acids protected from digestion within viral capsids and other small particles were then extracted using magnetic beads of MagMAX Viral RNA Isolation kit (Ambion) according to the manufacturer’s instructions. Reverse Transcription was then performed using a primer containing a fixed sequence followed by a randomized octomer at the 3′ end. A single round of DNA synthesis was then performed using Klenow fragment polymerase [18]. Twenty cycles of PCR amplification of nucleic acids was then performed using primers consisting of the fixed portions of the random primers. Then the PCR products purified, cloned into T-vector, and sequenced. The resulted sequences were searched in GenBank using BLASTx. Our searching results showed that three samples showed positive for mammalian viruses, including two samples positive for anellovirus and one samples positive for a putative novel gemycircularvirus. Although anelloviruses are endemic worldwide, their infections were not associated with particular disease [19]. Therefore, anelloviruses were not considered to be a causative agent of two cases of encephalitis in the present study. The other one samples included a 435 bp sequence which had the highest sequence homology to gemycircularviruses, and shared 45–58 % amino acid sequence identities with gemycircularviruses, suggesting this is a novel gemycircularvirus. To exclude the possibility of virus nucleic acid contamination from environments or reagents [20], the gemycircularvirus-positive CSF samples and two negative controls including one gemycircularvirus-negative CSF sample and an equal volume of PBS were re-extracted by MiniBest viral RNA/DNA extraction Kit (TaKaRa, Japan). PCR with nested primers specific to the 435 bp sequence was performed to detect the gemycircularvirus gene. Primers used here are Gmv435FO (5′-GGACGGTAGCGATGCTCGGC-3′) and Gmv435RO (5′-TCGCGATGGCGGAATTCACCT-3′) for the 1st round PCR, and Gmv435FI (5′-TGCTCGGCATTGTGTGAAGG-3′) and Gmv435RI (5′-ACACCATCCGAACACCAGCC-3′) for the 2nd round PCR. The PCR product size of the 2nd round PCR is about 250 bp. The specific DNA band was T-A cloned and sequencing result confirmed that the gemycircularvirus was present in the original positive CSF sample but not in the two control samples.

The genome sequences were then amplified by inverse PCR primers designed based on this 435 bp Rep fragment. The inverse primers are In435FP (5′-*G*CCCCCAGGCCTGCCCTTGCTA-3′) and In435RP (5′-*G*GGACCAGGAGAAGCTTCCAA-3′) for the 1st round PCR and In435FF (5′-GGGCTGGTGTTCGGATGGTGT-3′) and In435RF(5′-GCGGAGACTGGATCCTAGTGCGA-3′) for the 2nd round PCR. Here, the bases with asterisk means phosphorothioation. Primers’ position were shown in Fig. 1a. Sanger method was used for sequencing of the inverse PCR products. Our results indicated that the complete genome of the gemycircularvirus strain (named GeTz1; GenBank: KT363839) is 2202 bp in length, which exhibits the genomic features with a classic nonanucleotide motif of TAATATTAT nested within stem-loop structure similar to those found in geminiviruses, circoviruses, and nanoviruses [21–23]. The genome of GeTz1 contains two bidirectional genes encoding the Rep on the negative strand and the capsid protein (Cap) on the positive strand (Fig. 1a). An intron lies within the rep gene, which is similar to those in some geminiviruses [11, 24].

**Fig. 1:** Genome organization (**a**) and amino acid-based neighbor-joining analysis of Gemycircularvirus GeTz1(**b**). Phylogenetic tree was constructed with Mega5.0 from multiple alignments of the Rep proteins of the GeTz1 in the present study and other 27 representative gemycircularvirus strains from GenBanK. Two representative strains of geminivirus, nanovirus, cyclovirus and circovirus, respectively, were included as outgroup. Bootstrap values less than 70 were not shown. The scale bar indicates the number of substitutions per position for a unit branch length. Included with each taxa is the isolation source in which each sequence was found

To determine the relationship between GeTz1 in the present study and other gemycircularviruses in GenBank including those best maches of GeTz1 when performing BLASTx search, an alignment of Rep amino acid sequences was alignment was performed using CLUSTAL W (version 2.1) with the default settings [25]. A phylogenetic tree (Fig. 1b) with 100 bootstrap resamples of the alignment data sets was generated using the neighbor-joining method based on the Jones-Taylor-Thornton matrix-based model in MEGA5.0 [26]. Results indicates that GeTz1 clusters with one gemycircularviruses discovered from bird (KF371633) [8] sharing 46.6 % identity based on the complete amino acid sequence of Rep, which confirms GeTz1 belongs to a novel gemycircularvirus. Comparing with the other gemycircularvirus strain (SL1, NC_026818) isolated from CSF of a patients with encephalitis [3], GeTz1 shared 46.1 % sequence identity with SL1 over the complete Rep protein sequence.

To investigate the prevalence of this novel gemycircularvirus, primers described above (Gmv435FO, Gmv435RO, Gmv435FI, and Gmv435RI) were used to detect gemycircularvirus in 110 CSF samples collected from children (<6 years) with encephalitis. Result indicates all the samples are negative, which suggests that this novel gemycircularvirus strain is not prevalent in the children with encephalitis in this area.

Taken together, we describe a novel genome of gemycircularvirus in CSF from unexplained cases of encephalitis in China, which supports the possibility of replication of gemycircularvirus in the human host, however, data confirming replication of gemycircularvirus in mammalian cells or of sero-conversion to this virus are still lacking. Due to damage of labels during transportation and processing, we can only confirm that these CSF samples were from 20 samples with unexplained encephalitis, but we were unable to match clinical data with each individual samples. The detection of gemycircularvirus genome in mammalian feces, blood, and CSF [3, 8, 15], may reflect genuine viral replication in humans or alternatively fungal infection releasing virus into the blood stream, fungi or fungi-infected plants in the diet, contamination from the surface of the skin during phlebotomy, or even contamination from particles floating in air. Further studies should be performed to elucidate that whether gemycircularviruses are associated with diseases of humans and animals. Although no virus isolation was tried in this study, we are in the process of establishing a serological assay using recombinant Cap and Rep proteins.
